The article "Correlation of Clinicopathological Factors with Brain Tumor-Related Epilepsy in Glioma" was retracted in 2023. Reasons: unreliable results or conclusions; concerns about the data; concerns about the peer review; concerns about the citations.

# Correlation of Clinicopathological Factors with Brain Tumor-Related Epilepsy in Glioma

**DOI:** 10.1155/2022/4918294

**Published:** 2022-09-30

**Authors:** Zengliang Wang, Wensheng Yang, Yongxin Wang, Yirizhati Aili, Zhitao Wang, Quanyi Wang, Shunli Jiang, Guangning Zhang, Junchen Zhang, Bo Li

**Affiliations:** ^1^Department of Neurosurgery, First Affiliated Hospital of Xinjiang Medical University, Urumqi, Xinjiang, China; ^2^Department of Neurosurgery, Xinjiang Bazhou People's Hospital, Xinjiang, China; ^3^Department of Pathology, The Affiliated Chenggong Hospital of Xiamen University, Fujian, China; ^4^Department of Pathology, Affiliated Hospital of Jining Medical University, Jining, Shandong, China; ^5^Key Laboratory of Occupational Health and Environmental Medicine, Department of Public Health, Jining Medical University, Jining, Shandong, China; ^6^Department of Neurosurgery, Affiliated Hospital of Jining Medical University, Jining, Shandong, China

## Abstract

**Objectives:**

Glioma patients with brain tumor-related epilepsy (BTRE) have a complex profile due to the simultaneous presence of two pathologies, glioma and epilepsy; however, they have not traditionally received as much attention as those with more malignant brain tumors. The underlying pathophysiology of brain tumor-related epilepsy remains poorly understood. The purpose of this study was to investigate the possible correlation between molecular neuropathology and glioma with BTRE and a wide range of BTRE-associated molecular markers of glioma patients.

**Methods:**

A retrospective cohort study of 186 glioma patients was evaluated at our hospital, of which 64 had BTRE. The chi-square test, Spearman rank correlation, and multivariate logistic analyses were used to identify clinicopathological factors associated with BTRE in glioma patients.

**Results:**

Of the 186 patients examined in this study, 64 (34.4%) had BTRE. Based on the analysis of the characteristics of these patients, the results showed that patient age (over 40 years; *P* = 0.007), low WHO grade (grade I, II; *P* = 0.001), IDH-1 positive mutation (*P* = 0.027), low ATR-X expression level (OR = 0.44; 95% CI: 0.21, 0.92), and low Ki-67 PI (OR = 0.25; 95% CI: 0.10, 0.68) were associated with the occurrence of BTRE. In our cohort, BTRE patients did not differ by sex, tumor location, or expression of olig-2 and CD34. The results of the matching study showed that low Ki-67 PI and negative ATR-X expression levels were independent factors for a higher incidence of preoperative seizures in glioma patients.

**Conclusion:**

The current study updates existing information on genetic markers in gliomas with BTRE and explores the correlation of a wide range of clinicopathological factors and glioma patients with BTRE and suggests three putative biomarkers for BTRE: positive IDH1 mutation, low Ki-67 PI, and negative ATR-X expression. These factors may provide insights for developing a more thorough understanding of the pathogenesis of epilepsy and effective treatment strategies aimed at seizure control.

## 1. Introduction

Epilepsy associated with brain tumors is called brain tumor-related epilepsy (BTRE), and the International Union of Antiepileptics (ILAE) defines tumor-related epilepsy as a persistent tumor lesion in the brain that causes more than one seizure [1, 2]. As the main symptom of brain tumors, epilepsy seriously affects the quality of life of patients. As a common brain tumor, most gliomas are caused by epilepsy, especially in patients with low-grade gliomas [3]. The frequency of epilepsy in patients with brain tumors ranges from 30 to 100% depending on the tumor type [1, 3–5], and the proportion of patients with epilepsy as the first symptom of gliomas can be as high as 50%-80% [6, 7], some studies in China showed that the incidence of glioma-related epilepsy before surgery was 34.1%, and the incidence of glioma-related epilepsy after surgery was 19.4%, the incidence of both preoperative and postoperative glioma-associated epilepsy was highest in anaplastic oligodendroglioma (AO) and lowest in IDH wild-type glioblastoma (GBM), and, patients less than 45 years old, with normal neurological function and lower WHO grade were more likely to have glioma-related epilepsy [8–10]. Although surgical resection of the tumor can improve the prognosis of epilepsy, there are still a small number of patients after surgical treatment who will still require drugs that have difficulty controlling epilepsy, known as refractory epilepsy [11, 12]. As the most common presentation of glioma and one of the main clinical symptoms in the early stage of glioma, epileptic seizures are also one of the most common reasons that many glioma patients visit the clinic for the first time, and most patients are diagnosed with gliomas due to seizures, which are often considered an early warning sign for glioma patients [13–16]. Both epileptic seizures and the use of antiepileptic drugs can lead to cognitive impairment in patients, and more than 10% of glioma patients will develop epileptic persistence. Despite various antitumor treatments, one-half of the patients had a seizure within 1 month and two-thirds within 3 months before the last evaluation, which affects their long-term quality of life and the therapeutic effect of glioma [7]. Also, numerous studies had shown that epilepsy was significantly associated with survival in patients with glioma, some studies found that postoperative glioma-associated epilepsy – but not preoperative glioma-associated epilepsy, predicted longer overall survival [8–10]. Therefore, a better understanding of BTRE's associated risks and production mechanisms can help to better predict, prevent, and control the occurrence of epilepsy, which is also of great significance for the comprehensive intervention of glioma patients.

The mechanism of brain tumor-related epilepsy is currently believed to be related to the tumor mass effect [17], formation of intracranial hypersensitized areas [18], local microenvironment changes in surrounding tumor tissues [19], and activation of the glutamate NMDA receptor [3]. Some studies have found that patients have extremely excited epileptogenic foci in the brain, including tumor cells and surrounding adjacent tissues caused by tumor compression or stimulation, and they can disrupt the brain's balance between excitement and inhibition by altering the expression of neuropeptides, neurotransmitters, and their receptors [3, 19]. In addition, the regional destruction of nerve cells in tumor cells and adjacent tissues leads to the blocking of afferent nerves in some cortical areas, which promotes the formation of an epileptogenic environment and the gradual development of a highly sensitized area for epileptic seizures [16]. Other studies have shown that local microenvironmental changes in brain tumor surrounding tissues can also induce seizures, such as swelling, ischemia, hypoxia, and acidosis. The depolarization and repolarization of ion channels on the cell membrane are unbalanced, which destroys the equilibrium of the local microenvironment of Na^+^, Ca^2+^_,_ and Cl^−^ plasma; increases the excitability of neurons, making them more vulnerable to external stimulation, and produces sudden, temporary abnormal discharge of neurons, leading to seizures. Studies have also shown that the NMDA receptor (N-methyl-d-aspartic acid receptor, or N-methyl-D-aspartate receptor) of glutamate can activate intracellular mTOR, AKT, MAPK, and other signaling pathways, leading to an increase in the frequency of epileptic seizures and a faster growth rate of tumor cells [3, 20, 21].

Previous studies have shown that the risk of seizures decreases with age, and that men are at higher risk than women. Additionally, tumor location (frontal, temporal, cap, pillow, island) and WHO classification (grades I ~ IV) are associated with brain tumor-related epilepsy [22, 23]. The incidence of brain tumor-related epilepsy in the frontal lobe, temporal lobe, insular lobe, and parietal lobe was higher than that in deep tumor tissues [24]. In summary, the pathophysiological mechanisms of brain tumor-related epilepsy are numerous and very complex, and there is no consensus on the effect of histopathological types and biomarkers on epilepsy risk. The correlation between IDH1 mutation, WHO pathological grade, and glioma tumor-related epilepsy has become a research hot spot; however, most of these studies have looked at prognostic relevance and drug therapy. Our study retrospectively analyzed the clinical and molecular pathologic data of all glioma patients surgically resected and routinely pathologically confirmed in our hospital over a 3-year period to study the relationship between gender, age, location of occurrence, and different molecular pathological markers in the occurrence of brain tumor-related epilepsy in glioma patients. We hope to have a more systematic and comprehensive understanding of epilepsy in glioma patients and provide theoretical support for better improving the quality of life of glioma patients.

## 2. Patients and Methods

### 2.1. Patients and Examination

This was a retrospective cohort study. The study was approved by the institutional review board (approval number: 2022C210) and was conducted according to the guidelines in the Helsinki Declaration and its later amendments. The informed consent was waived owing to the retrospective nature of this study. All the patients in this study were selected as following: a total of 256 human glioma specimens were collected from the Affiliated Hospital of Jining Medical University from January 2017 to December 2019, which were resected by neurosurgery and preserved completely and were diagnosed as glioma by pathology. All cases had complete clinical, imaging, and pathological data. MRI was performed in all patients after hospitalization to determine the location, size, and proximity of the tumor and to determine the tumor involvement in the lobe. Histological classification was carried out according to the 2016 WHO standards for grading tumors of the central nervous system. There were a total of I ~ IV levels, and the histological types mainly included astrocytoma, oligodendroglioma, and glioblastoma. The diagnosis of epileptic seizures was based on the criteria established by the 2017 International League Against Epilepsy (ILAE), and semiological seizure classification was performed by preoperative evaluation. The exclusion criteria were as follows: (1) craniocerebral trauma; (2) congenital cerebral vascular malformation, such as arteriovenous malformation and cavernous hemangioma; (3) other intracranial tumors, such as meningiomas and brain metastases; (4) infectious diseases of the central nervous system; (5) primary epilepsy caused by congenital neurological diseases, such as cortical dysplasia; (6) febrile epilepsy, drug-induced epilepsy, and other epilepsy unrelated to intracranial tumors; (7) nonfirst operation, chemoradiotherapy, and other treatments. And, the research flow chart of this study was shown in Figure 1. There is a department in our hospital that specializes in the follow-up of discharged patients, however, it is inevitable that some patients will be lost to follow-up, because some patients are involved in China and they are reluctant to disclose the condition of patients after discharge, especially the patients who died after discharge.

### 2.2. Clinical Variables

Information was collected, including age, gender, epileptic seizure, lesion location, IDH-1 mutation, WHO classification, Ki-67 proliferation index, CD34 expression, GFAP expression, olig-2 expression, and ATR-X expression (Tables 1 and 2 for details). The diagnosis of epileptic seizures was evaluated and guided jointly by certified neurologists and neurosurgeons. MRI was performed for all patients, and the lesion site was evaluated by a certified radiologist.

### 2.3. Laboratory Testing

All glioma specimens were immunostained, including CD34, oligo-specific nuclear transcription factor (OLIg-2), ATRX, P53, proliferation index (KI-67), and glial fibrillary acidic protein (GFAP), and all of the above monoclonal antibodies were purchased from Beijing Zhongshan Jinqiao Biological Co. Ltd. Sanger sequencing was used to detect the IDH1 R132H mutation. Immunohistochemistry (SP) used the following method: paraffin sections were placed in the oven at 60°C for 1 hour to prevent defoliation. Samples were dewaxed and rinsed 3 times with double steaming water for 5 minutes; the slices were put into citric acid buffer solution with pH 6.0, put into a pressure cooker and heated to boiling in a water bath. After 2 minutes in the water bath, the slices were naturally cooled at room temperature for 30 minutes and rinsed 3 times with PBS for 5 minutes. Next, 3% hydrogen peroxide was added to inactivate endogenous peroxidase; the samples were left at room temperature for 5-10 minutes and rinsed 3 times with distilled water for 5 minutes. Normal goat serum blocking solution was added, and the samples were incubated at room temperature for 20 minutes, added to 1 : 150 diluted primary antibody, and refrigerated overnight at 4°C. The cells were rinsed 3 times with PBS for 5 min, dripped with biotin-labeled secondary antibody, left at room temperature for 20 minutes, and rinsed 3 times with PBS for 5 minutes. Streptomycin antibiotic protein-horseradish catalase complex working solution was added, and the samples were incubated at 37°C for 10-15 minutes and rinsed 4 times with PBS for 5 minutes. DAB color developing agent was added to control the color developing under the microscope. The samples were fully rinsed with tap water, hematlignin was redyed for 25 seconds, and 1% alcohol was differentiated for 50 seconds. Ammonia returned the samples to blue, the samples were fully rinsed with tap water, hematlignin was slightly redyed, and the final samples were dehydrated and transparent. Neutral gum was used as the seal tablet, and PBS was used as the negative control instead of primary antibody. All operations were carried out in strict accordance with the kit instructions.

The YCTY2050 pathological image analysis system was used for quantitative determination. Specimens subjected to immunohistochemistry were assigned a grade for the staining intensity based on qualitative observations by two independent observers. GFAP was brownish yellow and stained in the cytoplasm and cell membrane. ATRX, Ki-67, and P53 were brownish yellow or brown particles, and the staining sites were the nuclei. The staining sites of CD34-positive cells were mainly in the cell boundary and cytoplasm, and uniform yellow staining was observed in vascular endothelial cells. Olig-2 was brownish yellow, with nuclei and cytoplasm as the staining sites, mainly nuclei.

The immunostained sections were observed with microscopes under low and high magnification, and 5 visual fields were randomly selected under high magnification (400X) to count 1,000 tumor cells and calculate the percentage of positive cells. The determination criteria for the results were as follows: negative (−): the tumor tissues were not stained at all or the number of positive cells was less than 5%; weak positive (+): the number of positive cells in tumor tissues was 6%-25%; positive (++): the number of positive cells in tumor tissues was 25%-50%; strong positive (+++): the positive number of tumor tissues was more than 50%. For the convenience of statistics, weak positive and negative were classified as negative, while positive and strong positive were classified as positive. The Ki-67 proliferation index (PI) was defined as the percentage of immunoreactive tumor cell nuclei among the total number of cells. PI was evaluated as follows: the number of positive cells ≤ 5% was considered low PI; the number of positive cells 6-20% was considered medium PI; and the number of positive cells > 20% was considered high PI.

### 2.4. Statistical Analyses

The results were analyzed with SPSS, version 22.0 (SPSS Inc., Chicago, IL, USA). Descriptive statistical methods were used to analyze the demographic characteristics, tumor location distribution, and immunohistochemical indices of the subjects. The frequency and percentage were used to describe the categorical variables statistically, and the chi-square test was used to analyze whether the difference between the two groups was statistically significant. The Spearman rank correlation was used to analyze the correlation between the immunohistochemical index and glioma with epilepsy. Multiple logistic regression was used to analyze the association between immunohistochemical indices and the risk of glioma with epilepsy, and the OR value and 95% CI were used as effect estimates. *P* < 0.05 was considered to be significant.

## 3. Results

### 3.1. Descriptive Characteristics of Glioma Patients

A total of 256 patients with glioma were included. And, none of the patients died during hospitalization. A total of 226 patients were recorded after excluding 15 patients with cavernous hemangioma, 8 with disordered cortical neurons, 6 with glial hyperplasia and 1 with medulloblastoma. In addition, 40 patients were excluded due to unqualified specimens (insufficient tissue, damaged wax blocks). Finally, 186 patients were included (81 males and 105 females; age range, 4–73 years; median age, 50 years) (Figure 1). We divided all patients into two groups based on preoperative seizure status: the BTRE (brain tumor-related epilepsy) group and the NO BTRE group. In the BTRE group, there were 64 patients, including 34 males and 30 females, 23 (35.9%) under the age of 40 years and 41 (64.1%) over the age of 40 years. In the NO BTRE group, there were 122 patients, including 47 males and 75 females, 22 (18.0%) under the age of 40 years and 100 (82.0%) over the age of 40 years. Tumor location was analyzed using MRI characteristics, and the tumor side was not considered in this study to better define the correlation between molecular indicators and tumors related to epilepsy. The most commonly involved location was multiple lobes (*N* = 65, 34.9%), followed by the frontal lobe (*N* = 55, 29.6%), the temporal lobe (*N* = 44, 23.7%), the cerebellum (*N* = 7, 3.8%), the parietal lobe (*N* = 6, 3.2%), the basal ganglia region (*N* = 3, 1.6%), the thalamus and occipital lobe (*N* = 2, 1.1%), and the insula, and intraventricular regions (*N* = 1, 0.5%) (for details, see Tables 1 and 2). Since the focus of this study was on the correlation of clinicopathological factors with brain tumor-related epilepsy in glioma of the patients, the survival rate of patients was not counted, so patients who died or were lost to follow-up after discharge were not counted.

The pathological results showed that the BTRE group included 5 grade I, 35 grade II, 14 grade III, and 10 grade IV patients; the NO BTRE group included 7 grade I, 32 grade II, 40 grade III, and 43 grade IV patients. The baseline information of all patients is summarized in Table 2. All 186 patients were successfully collected and analyzed for the expression levels of GFAP, olig-2, ATR-X, CD34, and p53. IDH mutation and Ki-67 PI were also recorded and analyzed (Table 1). The histopathological type of all the patients was also collected and analyzed (2016 World Health Organization (WHO) Classification of Tumors of the Central Nervous System); see Table 2.

### 3.2. Main Results

To identify factors that might be associated with tumor-related epilepsy, demographic and tumor information was compared between patients with and without seizures (see Table 1 for a complete list). Demographic statistics showed that there were significantly more female (56.5%) glioma patients than male (43.5%) patients; however, males (53.1%) had a higher incidence of BTRE than females (46.9%). The chi-square test showed no statistical significance (*P* = 0.056). The statistical results showed that there were significantly more glioma patients older than 40 years than younger than 40 years, and the incidence of TRE in patients older than 40 years was significantly higher than that in patients younger than 40 years (*P* < 0.05). The statistical results of the correlation between tumor location and epilepsy showed that glioma tended to occur in multiple lobes (34.9%), followed by the frontal (29.6%) and temporal lobes (23.7%), while BTRE tended to occur in the frontal lobe (35.9%), followed by multiple (34.4%) and temporal lobes (23.4%), and the difference was not statistically significant (*P* = 0.594). The WHO classification results showed that TRE occurred mainly in patients with low-grade glioma (WHO grade II (54.7%)), followed by patients with high-grade glioma (WHO grade III (32.8%), WHO grade IV (35.2%)), and the difference was statistically significant (*P* < 0.05). Histopathological results showed that glioblastoma IDH wild-type (20.4%) and anaplastic astrocytoma IDH wild-type (17.7%) were lower in the NO BTRE group, diffuse astrocytoma IDH wild-type (23.4%) was higher in the TRE group, and the difference in tumor histological type between the two groups was statistically significant (*P* < 0.001); for details, see Table 2. Analysis of immunohistochemical indices and IDH1 mutation results showed that three variables were significantly associated with the presence of epilepsy: IDH-1 mutation (*P* = 0.027), low ATR-X expression level (*P* = 0.041), and low Ki-67 PI (*P* = 0.001) (Table 2). The Spearman rank correlation analysis showed that the correlation coefficient between IDH-1 mutation and BTRE was 0.16, with a significant positive correlation (*P* < 0.05). The correlation coefficients between ATR-X-positive expression and Ki-67 PI and BTRE were −0.17 and −0.28, respectively, and they were significantly negatively correlated with TRE (*P* < 0.05) (Table 3). Representative immunohistochemical staining for Ki-67 labeled from low to high (low, ≤5%; medium, 6-20%; high, >20%), ATR-X positive or negative expression and analysis of IDH1 mutation with negative and positive results are shown in Figures 2, 3, and 4, respectively. No other clinical or pathological variables were found to be associated with an increased risk for preoperative seizures in this group of patients. In the multinomial logistic regression analysis, after adjusting for gender, age, and WHO grade, the incidence of epilepsy in glioma patients with ATR-X-positive expression was significantly reduced (*P* = 0.029), and the risk was 56% lower than that in the ATR-X-negative expression group (OR = 0.44; 95% CI: 0.21, 0.92). Compared with that in the low-proliferation Ki-67 group, the incidence of epilepsy in glioma patients in the high-proliferation Ki-67 group was significantly reduced (*P* = 0.006), and the risk was reduced by 75% (OR = 0.25; 95% CI: 0.10, 0.68). That is, low Ki-67 PI and low ATR-X expression levels were found to have a strong association with preoperative seizures, which were independent factors for a higher incidence of preoperative seizures (Table 4).

## 4. Discussion

Brain tumor-related epilepsy (BTRE) is a type of epilepsy induced by the abnormal discharge of the intracranial tumor itself or its mass effect caused by the abnormal discharge of nerve cells around the lesion^1^. Seizures are one of the clinical symptoms of brain tumors, so patients can also present with disorders of consciousness, limb movement, and sensory and autonomic nervous function [25–27]. Seizures are often seen in patients with brain tumors and occur at different rates. However, there is no clear conclusion on the pathogenesis and pathophysiology of BTRE, and there is no single theory that can explain the cause of BTRE, which is a relatively complex and multifactor seizure [28–31].

Seizures and the use of antiepileptic drugs can lead to cognitive impairment, affect the long-term quality of life of patients, and have curative effects on brain tumors, which can also affect patients' family harmony, poor working conditions, and low moods [29]. Patients with brain tumor-related epilepsy (BTRE) present a complex therapeutic profile and require a unique and multidisciplinary approach. They, in fact, must face two different pathologies at the same time, brain tumor and epilepsy. In brain tumor patients, the presence of epilepsy is considered the most important risk factor for long-term disability [32, 33]. The problem of the proper administration of medications and their potential side effects is of great importance because good seizure control also has a significant impact on the patient's psychological and relational sphere [33]. Therefore, it is necessary to understand the mechanism of BTRE to better predict, prevent, and control the occurrence of epilepsy. With the progress of research methods and technologies, BTRE has been deeply explored, especially in terms of its pathogenesis and the corresponding brain neural network. However, there is still a lack of sufficient attention and systematic research on the pathogenesis, clinical diagnosis, and treatment of BTRE. At present, few studies have focused on the molecular neuropathologic correlation of glioma with tumor-related epilepsy [11], except for several studies on the association between WHO classification and IDH1 mutation in brain tumor-related epilepsy of patients with low-grade glioma [25, 34, 35]. Therefore, to better define the etiology of tumor-related epilepsy in glioma patients, our study focused on the correlation between molecular neuropathic indicators and BTRE in low and high glioma patients, which was expected to clarify the pathogenesis of glioma patients with BTRE and benefit glioma patients. This large cohort of glioma patients was treated at a single institute in China over a period of 3 years.

To our knowledge, this is the first systematic retrospective study to investigate the correlation between molecular neuropathology and different grades of glioma in patients with BTRE. In the 186 glioma patients, the results showed that patients aged over 40 years old and with a low WHO grade were significantly correlated with BTRE. Additionally, we identified one histopathological type and three molecular pathological characteristics that were specifically associated with BTRE: diffuse astrocytoma, IDH wild type, low Ki-67 PI, negative ATR-X expression, and IDH-1 positive mutation status. In addition, Ki-67 PI and ATR-X expression were independent factors correlated with a higher incidence of preoperative seizures. Future research should focus on identifying susceptibility candidate genes for BTRE in larger multicenter studies, including low- and high-grade gliomas with and without symptomatic seizures.

Previous studies have shown that age, sex, tumor location, histopathological type, and WHO grade were the influencing factors of glioma with BTRE, although the results of various reports were inconsistent [25, 36, 37]. At present, there is no agreement on the influence of age, sex, and histopathological type on the occurrence of epilepsy. One study showed that the risk was higher in men than in women, and the risk of seizure decreased with age; however, the results varied among different histopathological types [38]. Previous studies have shown that the most common gliomas associated with epilepsy are diffuse astrocytoma, oligodendroglioma, and pleomorphic xanthoastrocytoma [39]. According to the World Health Organization Classification, 2016 edition [40], gliomas are classified as diffuse gliomas (astrocytoma, oligodendroglioma, and glioblastoma) and circumscribed and low-grade gliomas (angiocentric glioma, pilocytic astrocytoma, subependymal giant cell astrocytoma, pleomorphic xanthoastrocytoma, pilomyxoid astrocytoma, ependymoma, myxopapillary ependymoma, and subependymoma). Some research results showed that most patients with angiocentric glioma were children and young people, with no significant gender difference, and epilepsy was the main clinical manifestation [22]; diffuse astrocytoma and oligodendroglial tumors were common in the cerebral hemisphere of young patients (frontal and temporal lobes were common), and epilepsy was one of the most common clinical symptoms [41]. These results showed that low-grade gliomas were more common in young adults and were more common in the supratentorial frontal and temporal lobes, with no gender difference, and epilepsy was one of the main clinical symptoms. However, the previous studies were not entirely consistent with our findings. Our statistical results showed that BTRE was higher in male glioma patients than in female patients, but the results were not statistically significant. The incidence of BTRE in glioma patients older than 40 years was higher than that in glioma patients younger than 40 years, and the results were statistically significant. In addition, the most common histological types of BTRE in our study were diffuse astrocytoma, IDH wildtype, followed by oligodendrogastrocytoma, NOS; glioblastoma, IDH wildtype; and diffuse astrocytoma, IDH mutant. The relationship between the location of the glioma and BTRE risk has been controversial. Gliomas can occur in any part of the brain; however, frontal, temporal, and parietal gliomas are the most likely to be associated with BTRE, while occipital and supratentinal gliomas are less likely to have BTRE [39]. Our results showed that BTRE was most likely to occur in gliomas involving the frontal lobe and multiple lobes (see Table 2). The frontal lobe, temporal lobe, and parietal lobe are closely related to human language, consciousness, and motor functions. Lesions in these areas could cause abnormal discharge of these brain functional areas, leading to epilepsy. If the glioma invades the cortical functional area, the incidence of epilepsy will be higher. However, statistical results showed that the occurrence of BTRE was not statistically significant in relation to the location of the tumor, which was different from previous studies [36]. The reasons for the different statistical results may be related to differences in study design and populations or the complex mechanism of BTRE, and the results of individual research centers could be different.

Previous studies have shown that seizures are more common in low-grade gliomas than in high-grade gliomas [1, 3]. The results were similar to those in our study, which showed that BTRE was present in lower grade gliomas at 62.5% and in higher grade gliomas at 37.5%. This may be related to the faster growth rate of high-grade glioma, which will cause severe ischemic and hypoxic damage to the surrounding tissues and tumor tissues themselves, making them less likely to form epileptogenic foci. Other studies have suggested that high-grade gliomas release excessive amounts of the neuroexcitatory transmitter glutamate, which is neurotoxic and can lead to neuronal death in large quantities, so high-grade gliomas are less likely to have seizures [42]. Some studies have also suggested that the rapid growth of high-grade gliomas destroys the brain's electrical transmission network; however, low-grade glioma has a slow growth rate and little influence on the surrounding tissues, presenting with gradual degeneration, causing partial cortical afferent nerve block, leading to high sensitivity of demulsification, and promoting the formation of epileptogenic foci [17, 43]. At present, the correlation and mechanism of BTRE in different WHO grade gliomas mainly focus on the destruction of the blood–brain barrier, gene mutations, changes in neurotransmitters, and receptors, and changes in ion concentration. Additionally, studies have shown that cellular inflammatory factors are involved in the occurrence and development of BTRE in glioma [44, 45]. Despite numerous studies, the mechanism of BTRE in different grades of gliomas is still unclear and needs further research.

Isocitrate dehydrogenase (IDH) is a member of the *α*-hydroxy acid oxidative decarboxylase family. IDH mainly acts on the tricarboxylic acid cycle to convert isocitrate into *α*-ketoglutaric acid, while the IDH mutation could convert isocitrate into 2-hydroxyglutaric acid (2-HG); the altered reaction is known as the weakening of alpha-ketoglutaric acid, which increases the level of 2-HG [46]. The IDH mutation was first identified in low-grade glioma patients, which was an early event in gliomagenesis and has significant implications for glioma progression and tumor behavior [47]. A previous study showed that mutation of the IDH gene occurred in ~80% of lower-grade (WHO grade II and grade III) gliomas [48]. Mutant IDH produces (R)-2-hydroxyglutarate, which induces DNA hypermethylation and presumably drives tumorigenesis, which also suggests that 2-HG plays an important role in the occurrence and development of epilepsy. Due to 2-HG being structurally similar to glutamate, IDH1 mutant glioma cells release a large amount of 2-HG that will combine multiple neurons and activate receptors, such as NMDARs and AMPARs, causing the influx of sodium ions, potassium ions, and calcium ions, increasing the action potential triggered by neurons, and damaging the balance between the inhibition and excitation of neurons, thus causing abnormal excitation of neurons and promoting the occurrence of epilepsy [49]. Therefore, the incidence of BTRE in IDH1 mutant glioma patients is much higher than that in IDH1 wild-type patients. Our study showed that the IDH1 positive mutation incidence in glioma patients with epilepsy was 23.4%, which was different from IDH1 negative mutation incidence in the NO BTRE group (13.9%), and the difference was statistically significant, which suggested that IDH1 positive mutation was closely related to BTRE in glioma patients. Our study also showed that IDH1 mutation was more likely to occur in diffuse astrocytoma patients.

In our study, we identified two important molecular pathological characteristics associated with BTRE in glioma patients: Ki-67 PI and ATR-X expression. Tumor-correlated biomarkers in glioma patients with BTRE have been a popular research topic for decades; however, they have not traditionally enjoyed as much attention as more malignant brain tumors. In recent years, a number of developments have been achieved toward further understanding the molecular and developmental backgrounds of glioma patients with BTRE, which helps to clarify the mechanism of glioma leading to epileptic seizures. Several studies have shown that a number of candidate genes cause seizures in glioma patients, such as interleukin-1*β* (IL-1*β*) [50], CD34 [51], and tuberous sclerosis complex (TSC) [52]. Molecular genetic effects may alter the balance between intracortical inhibitory and excitatory mechanisms, therefore inducing epileptogenic activity. However, the molecular mechanism underlying BTRE remains largely unknown, and there is still an issue of whether BTRE in glioma patients results from localized epileptic foci that lead to abnormal circuits or from molecular defects. Ki-67 is a protein found in the nucleus of a cell. Ki was discovered in the 1980s in Kiel, Germany, and the number 67 comes from the experiment number. Researchers have found a strong link between the amount of this protein and the cell division cycle; the higher the positive rate of Ki-67 is, the higher the proportion of cells in the proliferative cycle and the faster the tumor growth [53]. At present, Ki-67 has become a very important indicator to judge the activity level of tumor cells. The association between Ki-67 and BTRE in glioma patients has rarely been studied, and the results have been inconsistent [54]. One study showed that the Ki-67 proliferation index was not associated with the risk of epileptic seizures in glioma patients [55]. However, some studies have also suggested that Ki-67 significantly affects seizure prognosis [56] and is related to BTRE in glioma by increasing proliferation [56]. These results indicated that Ki-67 may play a role in epilepsy in glioma patients. Low Ki-67 PI is usually associated with benign tumors or low-grade glioma (WHO grade I, II), and our study already showed that WHO grade I or II was associated with BTRE in glioma patients (Table 2), which supports our hypothesis that it could increase the incidence of preoperative seizures in glioma patients. In our study, a low Ki-67 PI was clearly associated with BTRE in glioma, with statistical significance. Of course, the results of this study cannot be taken as the final result, and the correlation between Ki-67 PI and epilepsy in glioma patients need further study. The ATR-X gene is a pathogenic gene of X-linked *α* thalassemia/mental retardation syndrome located on the X chromosome and plays an important role in chromatin remodeling, genome, and maintenance of telomere stability [57]. Mutations in ATR-X have been identified in multiple tumor types; in 2011, Heaphy et al. found that ATR-X gene mutation existed in tumors of the central nervous system, and a series of subsequent studies confirmed that ATR-X gene mutation mainly occurred in diffuse astrocytoma [58]; in 2014, the consensus of the International Society of Neuropathology considered the deletion of the ATR-X gene as a characteristic molecular marker of diffuse astrocytoma [59]; in 2016, the World Health Organization (WHO) integrated IDH, TERT, 1P19Q, and other molecular markers into the histopathological diagnosis of glioma, promoting the accurate diagnosis of glioma [37]. Under the guidance of molecular typing, the accurate treatment of glioma has been a popular research topic in recent years. The ATR-X gene mutation can be used as a prognostic indicator for glioma patients. However, the association between ATR-X and epilepsy in glioma patients has not been described. Our study showed that compared with the epilepsy group, glioma patients with ATRX gene-positive mutations in the nonepileptic group were less likely to develop epilepsy, which was statistically significant (see Tables 3 and 4). In this study, positive expression of the ATR-X gene in glioma patients was significantly negatively correlated with concurrent tumor epilepsy (*P* < 0.05), which was shown to be an independent predictor for preoperative seizures in glioma patients. This finding has not been previously reported, and the mechanism needs to be confirmed by further research. Therefore, we expect and speculate that Ki-67 and ATR-X may become novel diagnostic or therapeutic targets for tumor-related epilepsy in glioma in the future.

In our study, we did not find that glioma patients with tumors of different lobes and positive or negative expression of olig-2 and CD34 were significantly likely to present with epilepsy. These results differ from previous studies and may be due to differences in the number of cases, methods, and mechanisms involved [51]. In addition, some limitations should be presented as follows. First, the project design of a small sample (*N* = 186) and single center cannot produce effective results. Second, only 64 glioma patients had epilepsy, leading to a relatively limited statistical power. Thus, the adjustment in logistic regression may be too extensive. Third, there were no data for other molecules, such as p53, EGFR amplification, and 1p/19q deletion, which should clarify their correlation with BTRE in glioma patients. Thus, further studies are needed to provide more evidence to identify molecular markers related to glioma with BTRE.

## 5. Conclusion

In summary, this retrospective study investigated new molecular pathologic indicators in glioma patients with BTRE. Low WHO grade, age over 40 years old, IDH1 positive mutation, and low Ki-67 PI and ATR-X negative expression were predictive of the likelihood of epilepsy occurring in glioma patients. Thus, some of these factors will be worthy of further research as possible therapeutic targets, which may provide insights into developing a more thorough understanding of the pathogenesis of epilepsy and aim to improve the long-term remission rate of epilepsy before and after surgery.

## Figures and Tables

**Figure 1:** Research flow chart.

**Figure 2:** Photomicrographs of tumor tissue stained for ATR-X: (a) negative expression, (b) positive expression, original magnification: x400.

**Figure 3:** Photomicrographs of tumor tissue stained for Ki-67 PI: (a) low Ki-67 PI (≤5%), (b) medium Ki-67 PI (6-20%), (c) high Ki-67 PI (>20%), original magnification: x400.

**Figure 4:** Sanger sequencing analysis of IDH1 R132H mutation with negative (a) and positive (b) (the red arrow) results.

**Table 1:** Basic characteristics and immunohistochemical indices of the study population. Of the 186 glioma patients, 56.5% were women and 75.8% were aged 40 or older. In terms of immunohistochemical indices, the positive rate of IDH-1 in the epileptic group was significantly higher than that in the nonepileptic group, but the positive rates of ATR-X and Ki-67 proliferation were significantly lower than those in the nonepileptic group (all *P* < 0.05).

Characteristics	Total cases (*N* = 186)	Cases with epilepsy (*N* = 64)	Cases without epilepsy (*N* = 122)	*P* value
Sex, *N* (%)				0.056
(i) Male	81 (43.5)	34 (53.1)	47 (38.5)	
(ii) Female	105 (56.5)	30 (46.9)	75 (61.5)	
Age, years, *N* (%)				**0.007**
(i) < 40	45 (24.2)	23 (35.9)	22 (18.0)	
(ii) ≥ 40	141 (75.8)	41 (64.1)	100 (82.0)	
Immunohistochemical indexes				
GFAP, *N* (%)				0.530
(i) (-)	2 (1.1)	0 (0.0)	2 (1.6)	
(ii) (+)	182 (97.8)	63 (98.4)	119 (97.5)	
Missing	2 (1.1)	1 (1.6)	1 (0.8)	
Olig-2, *N* (%)				0.942
(i) (-)	7 (3.8)	2 (3.1)	5 (4.1)	
(ii) (+)	167 (89.8)	58 (90.6)	109 (89.3)	
Missing	12 (6.5)	4 (6.3)	8 (6.6)	
IDH-1, *N* (%)				**0.027**
(i) (-)	133 (71.5)	38 (59.4)	95 (77.9)	
(ii) (+)	32 (17.2)	15 (23.4)	17 (13.9)	
Missing	21 (11.3)	11 (17.2)	10 (8.2)	
ATR-X, *N* (%)				**0.041**
(i) (-)	70 (37.6)	29 (45.3)	41 (33.6)	
(ii) (+)	93 (50.0)	24 (37.5)	69 (56.6)	
Missing	23 (12.4)	11 (17.2)	12 (9.8)	
Ki-67, *N* (%)				**0.001**
(i) Low	41 (22.0)	22 (34.4)	19 (15.6)	
(ii) Medium	73 (39.2)	28 (43.8)	45 (36.9)	
(iii) High	72 (38.7)	14 (21.9)	58 (47.5)	
CD34, *N* (%)				
(i) (-)	30 (16.1)	9 (14.1)	21 (17.2)	0.731
(ii) (+)	123 (66.1)	42 (65.6)	81 (66.4)	
Missing	33 (17.7)	13 (20.3)	20 (16.4)	

**Table 2:** Pathological grade, tumor location, and histopathological type of the study population. There was no significant difference in tumor location between the epileptic group and the nonepileptic group (*P* = 0.594). IDH wild-type glioblastoma and IDH wild-type anaplastic astrocytoma were lower in the epileptic group, while IDH wild-type diffuse astrocytoma was higher in the epileptic group, and the difference in tumor histological type between the two groups was statistically significant (*P* < 0.001). The WHO pathological grade of the epileptic group was mainly low grade, while that of the nonepileptic group was mainly high grade, and the difference was statistically significant (*P* < 0.001).

Characteristics	Total cases (*N* = 186)	Cases with epilepsy (*N* = 64)	Cases without epilepsy (*N* = 122)	*P* value
Pathological grade, *N* (%)				**0.001**
(i) Grade 1	12 (6.5)	5 (7.8)	7 (5.7)	
(ii) Grade 2	67 (36.0)	35 (54.7)	32 (26.2)	
(iii) Grade 3	54 (29.0)	14 (21.9)	40 (32.8)	
(iv) Grade 4	53 (28.5)	10 (15.6)	43 (35.2)	
Tumor location, *N* (%)				0.594
(i) Frontal	55 (29.6)	23 (35.9)	32 (26.2)	
(ii) Temporal	44 (23.7)	15 (23.4)	29 (23.8)	
(iii) Parietal	6 (3.2)	2 (3.1)	4 (3.3)	
(iv) Occipital	2 (1.1)	0 (0.0)	2 (1.6)	
(v) Insula	1 (0.5)	0 (0.0)	1 (0.8)	
(vi) Thalamus	2 (1.1)	1 (1.6)	1 (0.8)	
(vii) Cerebellar hemisphere	7 (3.8)	0 (0.0)	7 (5.7)	
(viii) Ventricle	1 (0.5)	0 (0.0)	1 (0.8)	
(ix) Basal ganglia	3 (1.6)	1 (1.6)	2 (1.6)	
(x) Multiple lobes	65 (34.9)	22 (34.4)	43 (35.2)	
Histopathological type, *N* (%)				<0.001
(i) Glioblastoma, IDH-wild type	38 (20.4)	7 (10.9)	31 (25.4)	
(ii) Diffuse astrocytoma, IDH-wild type	33 (17.7)	15 (23.4)	18 (14.8)	
(iii) Anaplastic astrocytoma, IDH-wild type	25 (13.4)	4 (6.3)	21 (17.2)	
(iv) Diffuse astrocytoma, IDH-mutant	11 (5.9)	6 (9.4)	5 (4.1)	
(v) Anaplastic oligodendroglioma, NOS	9 (4.8)	1 (1.6)	8 (6.6)	
(vi) Oligodendrocytoma, NOS	9 (4.8)	7 (10.9)	2 (1.6)	
(vii) Astrocytoma, NOS	8 (4.3)	4 (6.3)	4 (3.3)	
(viii) Oligodendroglioma, NOS	8 (4.3)	4 (6.3)	4 (3.3)	
(ix) Anaplastic astrocytoma, NOS	6 (3.2)	3 (4.7)	53 (2.5)	
(x) Glioblastoma, NOS	6 (3.2)	1 (1.6)	5 (4.1)	
(xi) Diffuse astrocytoma, NOS	6 (3.2)	4 (6.3)	2 (1.6)	
(xii) Pilocytic astrocytoma	5 (2.7)	0 (0.0)	5 (4.1)	
(xiii) Gliosarcoma	4 (2.2)	0 (0.0)	4 (3.3)	
(xiv) Anaplastic astrocytoma, NOS	3 (1.6)	1 (1.6)	2 (1.6)	
(xv) Glioblastoma, IDH-mutant	3 (1.6)	2 (3.1)	1 (0.8)	
(xvi) Pilomyxoid astrocytoma	2 (1.1)	1 (1.6)	1 (0.8)	
(xvii) Gemistocytic astrocytoma, IDH-wild type	1 (0.5)	1 (1.6)	0 (0.0)	
(xviii) Gemistocytic astrocytoma, IDH-mutant	1 (0.5)	0 (0.0)	1 (0.8)	
(xix) Anaplastic glioma, NOS	1 (0.5)	0 (0.0)	1 (0.8)	
(xx) Anaplastic pleomorphic xanthoastrocytoma	1 (0.5)	0 (0.0)	1 (0.8)	
(xxi) Anaplastic astrocytoma, IDH-mutant	1 (0.5)	0 (0.0)	1 (0.8)	
(xxii) Glial hyperplasia	1 (0.5)	1 (1.6)	0 (0.0)	
(xxiii) Ganglioglioma	1 (0.5)	1 (1.6)	0 (0.0)	
(xxiv) Diffuse glioma, NOS	1 (0.5)	0 (0.0)	1 (0.8)	
(xxv) Gangliocytoma	1 (0.5)	0 (0.0)	1 (0.8)	
(xxvi) Pilocytic astrocytoma	1 (0.5)	1 (1.6)	0 (0.0)	

**Table 3:** Spearman correlation coefficients among basic characteristics and tumor-related epilepsy. The Spearman correlation coefficient between the IDH-1 positive rate and tumor-related epilepsy was 0.16, with a significant positive correlation (*P* < 0.05). The Spearman correlation coefficients between the positive rate of ATR-X expression and the Ki-67 proliferation index and tumor-related epilepsy were −0.17 and −0.28, respectively, and they were significantly negatively correlated with tumor-related epilepsy (*P* < 0.05).

Variables	GFAP	Olig-2	IDH-1	ATR-X	Ki-67	CD34	Epilepsy
GFAP	1.00	0.25^∗∗^	0.05	–0.10	–0.12	0.16^∗^	0.08
Olig-2		1.00	0.01	–0.03	–0.07	0.13	0.03
IDH-1			1.00	–0.03	–0.19^∗^	–0.09	0.16^∗^
ATR-X				1.00	–0.004	0.04	–0.17^∗^
Ki-67					1.00	–0.07	–0.28^∗∗^
CD34						1.00	0.03
Epilepsy							1.00

^∗^ *P* < 0.05; ^∗∗^*P* < 0.001.

**Table 4:** Associations of immunohistochemical indices with the risk of having tumor-related epilepsy^a^. Multiple logistic regression was used to analyze the association between immunohistochemical indices and the risk of glioma complicated with epilepsy, and the results are shown in Table 4. After adjusting for gender, age, and WHO pathological grade, the incidence of epilepsy in patients with ATR-X-positive glioma was significantly reduced (*P* = 0.029), and the risk was 56% lower (OR = 0.44) than that in the ATR-X-negative group. 95% CI: 0.21, 0.92). Compared with the low-proliferation Ki-67 group, the incidence of epilepsy in glioma patients in the high-proliferation Ki-67 group was significantly reduced (*P* = 0.006), and the risk was reduced by 75% (OR = 0.25; 95% CI: 0.10, 0.68).

Variables		ORs (95% CIs)	*P* value
GPAF	(-)	1.00 (reference)	—
	(+)	0.31 (0.02, 5.09)	0.409

Oli-2	(-)	1.00 (reference)	—
	(+)	1.14 (0.32, 4.07)	0.840

IDH-1	(-)	1.00 (reference)	—
	(+)	2.30 (0.94, 5.63)	0.068

ATR-X	(-)	1.00 (reference)	—
	(+)	**0.44 (0.21, 0.92)**	**0.029**

Ki-67	Low	1.00 (reference)	—
	Medium	0.67 (0.27, 1.68)	0.394
	High	**0.25 (0.10, 0.68)**	**0.006**

CD34	(-)	1.00 (reference)	—
	(+)	0.86 (0.38, 1.96)	0.718

^a^Sex and age were adjusted in the model.

## Data Availability

The data used to support the findings of this study are included within the article.
